# Comparison of Two Sternal Closure Techniques Based on Risk Factors: A Prospective, Observational Study

**DOI:** 10.1155/2021/2169431

**Published:** 2021-10-08

**Authors:** Ali Cemal Duzgun, Ekin Ilkeli, Fehmi Katircioglu

**Affiliations:** ^1^Department of Cardiovascular Surgery, Ankara Training and Research Hospital, Ankara, Turkey; ^2^Department of Cardiovascular Surgery, Duzce State Hospital, Duzce, Turkey

## Abstract

**Background:**

Stainless steel wires are still commonly used as a sternum closure technique. However, it can cause fatal complications due to rupture and dehiscence. It was anticipated that the sternal Cable System (Pioneer Surgical Technology Inc., Marquette, MI, USA) could provide a better sternal fixation and reduce the possible complications. *Materials and Method*. A total of 100 patients (57 male, 43 female) at high risk of dehiscence were included in this prospective observational study. Among those with EuroSCORE value of 4 and above, patients with chronic lung disease, chronic kidney disease, diabetes mellitus, obesity, smoking, body mass index, advanced age, and resurgery were operated in two separate centers. Standard steel wires (*n*: 51) used for sternotomy were compared with the sternal cable (*n*: 49). Early and late sternal dehiscence rates were compared in the study. The relationship between risk factors causing dehiscence and both methods was assessed statistically.

**Results:**

Early dehiscence rates were 6.4% in those closed with a sternal cable (*n*: 3) and 11.8% in those closed with a sternal wire (*n*: 6) (*p* < 0.05)). In risky patients, body mass index was the most determining parameter in terms of sternum dehiscence risk.

**Conclusion:**

In risky patients, we recommend the sternal cable system as a good and reliable closure technique to achieve a more stable and compact sternum.

## 1. Introduction

Median sternotomy still continues to be the most common incision type in open heart surgery as an easy, safe, fast, and inexpensive method. It is easy to access to the heart and bigger vessels with this method. Although there are different techniques and methods for sternum closure, sternal closure with monofilament stainless steel wire is still the most commonly used method because it is inexpensive [1].

If adequate sternal closure could not be provided, complications can be fatal especially in patients with advanced age and comorbidities. It is important because of the high risk of sternal complications due to advanced age, chronic obstructive pulmonary disease (COPD), diabetes mellitus (DM), chronic renal failure (CRF), obesity, and osteoporosis. Rigid and strong fixation of the sternum also reduces the risk of complications.

The risk of developing infection after median sternotomy is between 0.2% and 10%, and morbidity and mortality rates vary between 5% and 25% in the presence of infection [2].

### 1.1. Study Hypothesis

In this prospective study, we compared the monofilament stainless steel sternum closure wire with the Sternal Cable System (Pioneer Surgical Technology Inc., Marquette, MI, USA) in patients operated by sternotomy. We tried to elaborate which factors are more predominant to create a safer technique to guide surgeons.

## 2. Materials and Method

A total of 100 patients (57 males, 43 females) who were scheduled to be operated in two tertiary stage cardiovascular surgery clinics between January 2017 and September 2019 in the same session were included in the study. Both groups included in the study were formed prospectively, two-centered. The same surgery team has conducted the operations in 2 different cardiovascular surgery centers. Exitus patients and patients who could not be followed up or out of follow-up were not included in the study. The data of 100 patients who were followed up regularly were evaluated. The study was carried out in parallel between the two centers in patients with risk factors determined in the same date range. The study was carried out on a certain number of patients, taking into account the sample size and the number of sternal cables available.

All groups have certain risk factors such as COPD, DM, CRF, advanced age, smoking, reoperation, and body mass index. BMI (body mass index) values of the patients were evaluated according to the American Centers for Disease Control and Prevention standards in three groups which are normal, overweight, and obese [3].

The demographic characteristics of the patients (age, gender, smoking, etc.), operation types (coronary, valve surgery, etc.), and complications (dehiscence, mediastinitis, revision, etc.) were recorded.

The reasons for using multifilament stainless steel cable and monofilament standard steel wires were recorded. Standard monofilament steel wires used in sternum closure were compared with multifilament stainless steel sternal cable.

### 2.1. Approach to Patients, Surgical Method, and Follow-Up

All patients were conducted median sternotomy. Shaving and skin cleansing was done 1 day before. The left internal mammary artery (LİMA) was removed unilaterally skeletonized. The sternum was closed in 51 of the patients who were operated by the same surgical team using sternal steel wire and the other 49 using a sternal cable. The sternotomies in both methods were closed in an 8-shaped fashion with 5 standard stainless steel wires and 1.0 mm multifilament stainless steel cable regardless of the length of the sternum.

The patients were followed up in terms of sternal dehiscence in the first 6 weeks (early period) and 6 months (late period). Sternal dehiscence grading was made according to a new classification which evaluates the anatomic changes and the condition of the pectoral muscle [4]. Patient data were collected and evaluated statistically.

This prospective study was reviewed and approved by the ethics committee, and informed consent was obtained from all enrolled patients. All patients were informed that the Sternal Cable System will be use (ethics committee: 05.11.2018-93471371-44/450-Ankara Training and Research Hospital).

### 2.2. Statistical Analysis

WEKA 3.6 and SPSS 11.5 software were used to evaluate the data. As descriptive, mean ± standard deviation and median (minimum-maximum) for quantitative variables, the number of patients (percentage) for qualitative variables was used.

In case of a difference between the categories of the qualitative variable with more than two categories in terms of the quantitative variable with Student *t*-test if normal distribution assumptions are met, if not, it was checked using the Mann–Whitney *U* test. Chi-square and Fisher exact tests were utilized to assess the relationship between two qualitative variables. Statistical significance level was set as 0.05. In the WEKA tool, logistic regression, multilayer perceptron, and J48 from classification methods were used. Since there are too many variables in the data set, the Info Gain Attribute Eval, Gain Ratio Attribute Eval, and Chi-Squared Attributed Eval methods in WEKA have been used to examine the importance of the variables and variables that were jointly identified as insignificant by the three methods and considered to be less important as clinical information were excluded from the data set.

A total of 7 variables (6 independent variables and 1 dependent variable) remained in the data set. These variables are gender, age, BMI, Lima use, smoking, comorbidity, and closure method. Percentages regarding the importance of the variable are given according to the closing method which is the dependent variable. The data set was evaluated using the 10-fold crossvalidation test option. Results of the outcome variable were given using accuracy, *F*-measure, precision, and recall as the evaluation criteria.

## 3. Results

The demographic data of the patients are presented in Table 1.

When both sternum closure techniques are compared, early dehiscence rates were 6.4% in cases closed with sternal cable and 11.8% in cases closed with sternal wire (*p* < 0.05) (Table 2).

Obesity, diabetes, age, and dehiscence were the most common reasons for using sternum cable or sternum wire (Table 3).

Hospitalization durations and drainage rates were found to be higher in patients who were closed with a sternal cable (*p* < 0.05) (Table 4).

There was no difference between the two groups in terms of sternum revision and sternal infection. Mediastinitis occurred in 3 patients with sternal cable. However, this ratio was not clinically significant since dehiscence and revisions (n: 4) were closed with a sternal cable.

Hospitalization durations were determined as, respectively, mean ± SS4.43 ± 3.16 − 2.73 ± 0.78 between the sternal cable and sternum wire groups.

The potential superiority of the Sternal Cable System was evaluated significantly in the gain chart graph of the multilayer perceptron method (Figure 1).

## 4. Discussion

In recent years, surgeries performed in cardiac operations with minimally invasive incision have provided a lot of comfort. However, it is difficult to reach to the entire mediastinum with a single incision. It is advantageous to reach and maneuver to the entire mediastinal space with an easy and inexpensive incision such as a median sternotomy. However, it continues to carry the risk of dehiscence.

Preoperative risk factors for sternal dehiscence were indicated as obesity, COPD, osteoporosis, heart failure (New York Heart Association functional class III–IV), corticosteroid, immunosuppression, diabetes mellitus, renal failure, and previous sternotomy [5, 6].

If sternal healing is not achieved well after median sternotomy, it causes sternal separation and sternal dehiscence, resulting in severe sternal complications between 0.5% and 2.5% [7, 8]. Sternal dehiscence may become in mediastinitis, osteomyelitis, and unstable sternum forms, resulting in mortality of 10% to 40% as a result [9, 10]. Sternal stability is very important in sternum closure. Dehiscence developing due to unstable sternum is the main cause of sternal wound infections. The movements caused by the inability to join the bones rigidly cause tissue necrosis by damaging the surrounding tissues, which facilitates bacterial growth. [11]

In a study comparing traditional sternum wiring and rigid sternum fixation techniques, it was stated that clinical stability was significantly better in subjects who underwent rigid fixation 4 weeks after the operation and bone formation occurred in the osteotomy space during this period [12].

Although many sternum closure techniques have been reported, there is no consensus on the ideal closure technique. Multifilament Stainless Cable System (Pioneer Surgical Technology Inc. Marquette, MI, USA) is a model designed to be used in sternum closure. Previously, it was reported that the failure rate of the sternum cable after implantation was lower than the sternum wire and plates in a study comparing the sternum cable, sternum wire, and sternal plates used for sternum closure as form of eight [13]. According to this study, metal fatigue caused by the force to separate the two halves of the sternum and the associated implant failure risk is significantly lower in the cable system compared to the wire and plate.

As a result of this test separating the sternum from each other repeated 7.8 million times, there are no error lines on the curve showing the cables, and the success rate is 100%. Another test performed by applying opposite forces on the vertical axis to shift the two connecting parts of the sternum is 10,000 times showed that almost all of the traditional sternum wires were damaged (<0.001%) while 99.5% of the sternal cables continued the test without any damage. The performance of the plates is also lower than the sternal cable [14].

Multifilament cable wiring system has been stated to have about ten times stronger durability than standard steel wires [15]. The tensioning and compression tool used to close the sternum with the sternal cable allows the cable to be stretched in a controlled manner after the cable is placed in the sternum (the most effective application is the intercostal placement in the form of eight). The tension of the cable and thus the force applied to the sternum can be followed up from the indicator on the instrument. This feature ensures that each cable placed in the sternum is covered with the same tension and distributes the pressure homogeneously over the sternum (Figure 2). It distributes the pressure homogeneously over the sternum that occurs when the patient is breathing, coughing, or sneezing. Tightening the sternum at different points with equal strength also increases stabilization.

Since there is no possibility to adjust the pressure in the placement of traditional sternum wires, if the sternum is tightened with unequal forces at different points, all the resulting force due to the abovementioned reasons may overlap on the tightest ring and cause implant failure, the wire to cut the bone, or sternum fractures.

Particularly, since the bone compression procedure is adjusted by the surgeon in the sternal cable method, the equal and homogeneous distribution of pressure provides decrease in complications in CRF, COPD, DM, and osteoporotic patients.

Multifilament Stainless Cable Closure System produced more successful results in early dehiscence rates. The difference between sternal cable and sternal wire was detected as 3 6.4% and 11.8%, respectively (*p* < 0.05). This result means cost reduction as well as patient health. There was no statistically significant difference between the two groups in late dehiscence development.

Sternal bleeding is an important cause of drainage in most patients [16]. Higher drainage rates are related to patient characteristics rather than the Sternal Cable System. No clinically significant drainage was found. We found that the type of operation performed (aortic valve replacement, mitral valve replacement, coronary bypass, aortic surgery) did not make any difference in dehiscence formation. In a prospective, observational study performed on diabetic patients who are in risky patient group, sternal weave closure technique has been shown to be superior to standard sternum closure. [17]

No new approach has been developed for risky patient groups. One of the results of our study was to contribute to the creation of a strategy for the application of methods such as the Multifilament Stainless Cable Closure System, which is an alternative to the standard closure technique; although, there are different techniques in the sternum closure process. In this manner, it was observed that the most basic invariant parameter was BMI when the data is analyzed. Comorbidities have been another important determining parameter. Age, Lima use, and smoking were among the other determinants. Other risks that have formed the basic parameters and the strategy were overweight, use of sternal cable in women, and over 80 years old men, obviously, and seem to be more advantageous. In our experience, sternal dehiscence developed in the majority of patients while still in hospital or a few days after leaving the hospital. In our study, importantly, early dehiscence rates were found to be significantly lower in the sternal group compared to the wire group. Thus, fatal complications such as mediastinitis caused by dehiscence can be prevented in risky patient groups. We think that this will contribute to the recognition of risk factors and the strategy to be developed. While it should not be used for every patient, it will be particularly beneficial for patients over 80 years of age, osteoporotic, smoking, and with high BMI and where Lima will be used as a graft. We think that it is essential to develop a treatment strategy with a cable in these patients.

### 4.1. Limitations of the Study

The main limitation of our study is the limited number of patients in only two centers, because sufficient financial resources and time could not be provided. Therefore, multicentered, comprehensive, randomized studies may provide better results. More comprehensive studies are needed regarding which patients should be approached with which strategy.

It is possible to develop this basal strategy and to separate the risk groups, add additional recommendations, or add different surgical procedures (such as minimally invasive, pectoralis major flap) in patients with high dehiscence risk.

## 5. Conclusion

We recommend multifilament stainless cables as a good and reliable closure technique for a more stable and compact sternum in risky patients. BMI in particular, advanced age, Lima use, being overweight, smoking, and female gender have attracted attention as an important baseline parameter in the development of strategy in patients who may have sternum dehiscence risk.

## Figures and Tables

**Figure 1:** Tree diagram of J48 method and ratios of variables.

**Figure 2:** Intraoperative image multifilament cable wiring system (the force applied to the sternum can be followed by the indicator on the instrument. This feature ensures that each cable placed in the sternum is closed at the same tension and distributes the pressure homogeneously over the sternum).

**Table 1:** Demographic characteristics of the patients.

Variables	Groups			
	Sternal cable		Sternum wire	
	*n*	%	*n*	%
Gender				
Male	30	61.2	27	52.9
Female	19	38.8	24	47.1
Age				
<80	38	77.6	41	80.4
≥80	11	22.4	10	19.6
BMI				
Normal	13	27.7	17	33.3
Overweight	22	46.8	15	29.4
Obese	12	25.5	19	27.3
Smoking				
No	27	57.4	30	58.8
Yes	20	42.6	21	41.2

**Table 2:** Intraoperative and postoperative results.

Surgery	CABG	30	61.2	36	70.6
	AVR	3	6.1	4	7.8
	MVR	7	14.3	6	11.8
	CABG+MVR	5	10.2	3	5.9
	Aortic aneurisym dissection	2	4.1	2	3.9
	CABG+AVR	2	4.1	0	0.0

Lima usage	No	20	42.6	24	48.0
	Yes	27	57.4	26	52.0

Early dehiscence	No	44	93.6	45	88.2
	Yes	3	6.4	6	11.8

Late dehiscence	No	48	98.0	49	96.1
	Yes	1	2.0	2	3.9

Str. revision	No	40	81.6	43	84.3
	Yes	9	18.4	8	15.7

Str. infection	No	45	91.8	47	92.2
	Yes	4	8.2	4	7.8

Mediastinitis	No	45	93.8	50	98.0
	Yes	3	6.2	1	2.0

Death	Alive	46	93.9	51	100.0
	Death	3	6.1	0	0.0
	No	2	4.1	0	0.0

Str: sternal.

**Table 3:** Sternal cable and sternum wire usage reasons.

Reasons	Sternal cable		Sternal wire	
	*n*	%	*n*	%
Dehiscence	3	6.1	0	0.0
Older age	11	22.5	10	19.6
CRF	7	14.4	3	5.9
COPD	6	12.2	10	19.6
Obesity-DM	11	22.4	19	37.3
Reoper	8	16.3	9	17.6
Revision	1	2.0	0	0.0
Other	2	4.1	0	0.0

**Table 4:** Comparison of groups.

Variables	Groups					
	Sternal cable			Sternal wire		
	*n*	Mean ± SD	Median (min.-max.)	*n*	Mean ± SD	Median (min.-max.)
Intensive care stay	49	4.43 ± 3.16	3.00 (1.00-17.00)	51	2.73 ± 0.78	3.00 (2.00-6.00)
Hospital stay	49	8.41 ± 4.61	7.00 (2.00-27.00)	51	7.88 ± 2.36	7.00 (5.00-15.00)
Drainage	49	1033.47 ± 527.25	900.00 (15.00-2400.00)	51	739.22 ± 244.61	750.00 (350.00-1300.00)
Pain killer requirement	44	2.39 ± 1.15	2.00 (1.00-6.00)	50	1.98 ± 0.89	2.00 (1.00-4.00)
Age	49	66.55 ± 13.24	67.00 (22.00-86.00)	51	67.75 ± 9.18	68.00 (52.00-85.00)
BMI	47	27.44 ± 4.04	26.40 (21.40-36.35)	51	28.69 ± 4.74	26.40 (22.84-37.83)

## Data Availability

Data is available and can be sent at any time if requested by the journal editorial.
